This article has been retracted.

# LncRNA AATBC regulates Pinin to promote metastasis in nasopharyngeal carcinoma

**DOI:** 10.1002/1878-0261.12703

**Published:** 2020-06-13

**Authors:** Ting Tang, Liting Yang, Yujian Cao, Maonan Wang, Shanshan Zhang, Zhaojian Gong, Fang Xiong, Yi He, Yujuan Zhou, Qianjin Liao, Bo Xiang, Ming Zhou, Can Guo, Xiaoling Li, Yong Li, Wei Xiong, Guiyuan Li, Zhaoyang Zeng

**Affiliations:** ^1^ NHC Key Laboratory of Carcinogenesis and Hunan Key Laboratory of Translational Radiation Oncology Hunan Cancer Hospital and the Affiliated Cancer Hospital of Xiangya School of Medicine Central South University Changsha China; ^2^ Key Laboratory of Carcinogenesis and Cancer Invasion of the Chinese Ministry of Education Cancer Research Institute Central South University Changsha China; ^3^ Department of Stomatology Xiangya Hospital Central South University Changsha China; ^4^ Department of Oral and Maxillofacial Surgery The Second Xiangya Hospital Central South University Changsha China; ^5^ Department of Medicine Comprehensive Cancer Center Baylor College of Medicine Houston TX USA

**Keywords:** apoptosis‐associated transcript in bladder cancer, metastasis, miR‐1237‐3p, nasopharyngeal carcinoma, pinin, ZEB1

## Abstract

Long noncoding RNA (lncRNA) have emerged as crucial regulators for a myriad of biological processes, and perturbations in their cellular expression levels have often been associated with cancer pathogenesis. In this study, we identified AATBC (apoptosis‐associated transcript in bladder cancer, LOC284837) as a novel lncRNA. AATBC was found to be highly expressed in nasopharyngeal carcinoma (NPC), and increased AATBC expression was associated with poor survival in patients with NPC. Furthermore, AATBC promoted migration and invasion of NPC cells *in vitro,* as well as metastasis *in vivo*. AATBC upregulated the expression of the desmosome‐associated protein pinin (PNN) through miR‐1237‐3p sponging. In turn, PNN interacted with the epithelial–mesenchymal transition (EMT) activator ZEB1 and upregulated ZEB1 expression to promote EMT in NPC cells. Collectively, our results indicate that AATBC promotes NPC progression through the miR‐1237‐3p–PNN–ZEB1 axis. Our findings indicate AATBC as a potential prognostic biomarker or therapeutic target in NPC.

## Graphical abstract

Tang *et al*. found a novel lncRNA, AATBC, was upregulated in nasopharyngeal carcinoma (NPC) and associated with poor prognosis. Moreover, *in vitro* and *in vivo* experiments confirmed that AATBC promoted migration and invasion of NPC cells through sponging miR‐1237‐3p and upregulating PNN. In turn, PNN interacted with the ZEB1 and activated epithelial–mesenchymal transition in NPC cells.

**Abbreviations**
AATBC: apoptosis‐associated transcript in bladder cancer
ceRNA: competitive endogenous RNA
EMT: epithelial–mesenchymal transition
ISH: *In situ* hybridization
LC‐MS/MS: liquid chromatography‐tandem mass spectrometry
LncRNA: long noncoding RNA
MT: mutant type
NPC: nasopharyngeal carcinoma
NPE: normal nasopharyngeal epithelia
PNN: pinin
WT: wild‐type

## 1 Introduction

Nasopharyngeal carcinoma (NPC) is one of the most common cancers in southeastern provinces of China (Wei *et al*., 2017, Wu *et al*., 2019a, Zhao *et al*., 2020). Its epidemiology is characterized by its geographical distribution and ethnicity of these inhabitants. Genetic susceptibility, environmental factors, and Epstein–Barr virus infection play a significant role in carcinogenesis of NPC (Fan *et al*., 2018; Mo *et al*., 2019a; Tu *et al*., 2018, 2017; Xiong *et al*., 2004; Zeng *et al*., 2014, 2011, 2006). Although NPC is sensitive to radiotherapy with adjuvant chemotherapy (Ge *et al*., 2020; He *et al*., 2018; Tang *et al*., 2018a), most NPC patients often have metastases at the time of diagnosis. Hence, the prognosis of these patients is poor (Fan *et al*., 2019b; Peng *et al*., 2019; Ren *et al*. 2020; Wang *et al*., 2019a; Wei *et al*., 2018a, 2018b,2018a, 2018b; Xiong *et al*., 2019).

Long noncoding RNA (LncRNA) are transcripts longer than 200 nucleotides, which lack or possess no coding potential (Bo *et al*., 2019; Wang *et al*., 2020; Wei *et al*., 2019). LncRNA regulate gene expression through multiple mechanisms, and increasing evidence suggests their critical functions in cancer progression (Jiang *et al*., 2018; Jin *et al*., 2019; Liang *et al*., 2019; Wang *et al*., 2018). Intriguingly, recent studies have reported that some lncRNA function as ‘miRNA sponges’ or competitive endogenous RNA (ceRNA) to sequester miRNA and regulate their target mRNA (Wang *et al*., 2019b).

In this study, we found that the lncRNA, apoptosis‐associated transcript in bladder cancer (AATBC, LOC284837), was highly expressed in NPC and associated with poor prognosis of NPC patients. More importantly, AATBC acted as a ceRNA of PNN gene through competitively binding with miR‐1237‐3p. PNN promoted the epithelial–mesenchymal transition (EMT) progress through interacting with ZEB1, ultimately leading to metastasis of NPC.

## 2 Materials and methods

### 2.1 Tissues

Two sets of NPC samples were obtained from the Affiliated Cancer Hospital of Xiangya School of Medicine, Central South University, Hunan, China, for the study. Set 1 containing 18 NPC biopsies and 10 nasopharyngeal epithelial (NPE) tissues was used to analyze AATBC expression by qRT‐PCR. Set 2 containing 101 NPC and 34 noncancer NPE tissues was used to analyze AATBC expression for *in situ* hybridization (ISH) (Table S1). All the samples were confirmed by histopathological examination and handled according to the ethical and legal standards. The study was approved by the Research Ethics Committee of the Affiliated Cancer Hospital of Xiangya School of Medicine, Central South University, and the study methodologies conformed to the standards set by the Declaration of Helsinki. All patients who enrolled in the study signed the informed consent.

### 2.2 Cell culture, plasmids, and transfection

Nasopharyngeal carcinoma cell lines, 5‐8F, HNE2, and CNE2, were cultured in a humidified incubator under 5% CO_2_ at 37 °C. The cells were grown in RPMI 1640 medium supplemented with 10% FBS (Invitrogen, Shanghai, China), penicillin (100 U·mL^−1^; Sigma, St Louis, MO, USA), and streptomycin (100 µg·mL^−1^).

To overexpress AATBC, the full‐length AATBC coding sequence was cloned into a pcDNA3.1 plasmid. For PNN overexpression, the empty vector plasmid pCMV3‐C‐Flag (CV012) and the overexpression vector pCMV3‐PNN‐Flag (HG19349‐CF) were purchased from Sino Biological (Beijing, China). Sequences of AATBC and PNN siRNA are shown in Table S2. The mimics and inhibitors of miR‐1237‐3p were purchased from Ruibo Co (Guangzhou, China). For siRNA or miRNA transfection, cells were seeded and incubated overnight to perform transfection using Hiperfect Reagent (Qiagen, Hilden, Germany). For plasmid transfection, Lipofectamine 3000 (Invitrogen, Breda, the Netherlands) was used following the manufacturer's protocol.

### 2.3 RNA isolation and real‐time PCR

Total RNA from cell lines or tissues was isolated using Trizol reagent (Invitrogen, Carlsbad, CA, USA). The 5× all‐in‐one RT MasterMix kit (Applied Biological Materials, Richmond, BC, Canada) and gene‐specific or random primers were used in qRT‐PCR assay. SYBR^®^Green (Applied Biological Materials) was used for qRT‐PCR analysis performed in the MiniOpticon system (Bio‐Rad, Hercules, CA, USA). GAPDH and U6 snRNA were used as endogenous controls for mRNA/lncRNA and miRNA, respectively. Comparative *C*_t_ was used to calculate the relative expression of RNA. Primer sequences are listed in Table S2. For all qPCR assays using mRNA from cell lines, we used three technical replicates per sample and a representative image from two to three independent experiments was shown.

### 2.4 Transwell invasion assay

Transwell invasion assay was performed in 24‐well plates using the transwell (Corning, NY, USA) and Matrigel (BD Biosciences, San Jose, CA, USA) according to the manufacturer's instructions. A total of 1 × 10^5^ cells in 200 μL of serum‐free medium were added into the upper compartment of the chamber, and 800 μL of 20% FBS in the growth medium was added to the bottom well. After 36 h of incubation at 37 °C under 5% CO_2_, the cells invading through the Matrigel were fixed with methanol, stained with hematoxylin, and counted under a microscope. For each experiment, the number of cells invading Matrigel was counted from five visual regions randomly selected from the center and peripheral portions of the filter (Chen *et al*., 2019).

### 2.5 Scrape migration assay

Nasopharyngeal carcinoma cell lines, 5‐8F, HNE2, and CNE2, were inoculated and grown to 90% confluence in a 6‐well culture plate. The scratch was done by scraping the cell monolayers with a sterile 10‐μL pipette tip, and the scratch area was photographed by Leica DMI3000B computer‐assisted microscope (Leica, Oskar, Germany) at 100× magnification. Images were captured at 0, 12, and 24 h after the scratch. image‐pro plus 6.0 software (Media Cybernetics, Rockville, MD, USA) was used for image analysis (Cai *et al*., 2019).

### 2.6 Three‐dimensional (3D) invasion assay

Matrigel (BD Biosciences, San Jose, CA, USA) was melted at 4 °C after which 100 μL was added to each well of a 24‐well plate to cover the bottom of the plate. Plates were then incubated at 37 °C in a 5% humidified CO_2_ atmosphere for 1 h, and 0.1 mL of the cell suspension in culture medium containing 1 × 10^4^ cells·mL^−1^ was directly seeded into each well and incubated for 1 h. Next, Matrigel was diluted to a final concentration of 10% with RPMI supplemented with 10% FBS, which was added to the upper layer. After 2 days, the 300‐μL medium was replaced and cell morphology images were recorded for six consecutive days. The invasive degree of globules was of two types: noninvasive spheroids with smooth edges and no obvious cellular protrusions, or occasionally small scattered processes, and invasive spheroids containing fully scattered protrusions (Liu *et al*., 2019).

### 2.7 *In situ* hybridization

*In situ* hybridization was performed using three different nucleotide probes designed from different regions of AATBC. Three GAPDH probes were used as positive controls, and the probe sequences are shown in Table S2. Paraffin‐embedded sections were dewaxed at 80 °C and then were washed with 100% ethanol, 95% ethanol, 75% ethanol, 50% ethanol, and enzyme‐free water at 25 °C for 5 min each time. Then, the samples were treated with 3% hydrogen peroxide and fixed in 4% paraformaldehyde for 10 min, and digested in pepsin containing 3% citric acid, and then, the slides and probes were incubated with hybridization solution for 3 h at 37 °C before hybridization. The sections were incubated with anti‐AATBC oligodeoxynucleotide probe that was conjugated with antidigoxin at 37 °C humidified chamber for 16 h. After hybridization, the sections were washed in 1× PBS for 5 min and stained with hematoxylin (DAB, ZSGB‐BIO, Beijing, China). The staining intensity was according to the methods previously published (Zeng *et al*., 2007).

### 2.8 Animal studies

Eighteen 4‐week‐old nude mice obtained from the laboratory animal department of Central South University (Changsha, China) were randomly divided into three groups (*n* = 6 for each group) and maintained in a pathogen‐free environment. About 1 × 10^6^ 5‐8F cells transfected individually with negative control (NC), siAATBC, or the AATBC overexpression plasmid in 1× PBS were injected into the tail vein of the nude mice. After 8 weeks of injection, the mice were sacrificed, and the intact lung tissues were isolated, weighed, photographed, embedded in 10% paraffin, and stained with hematoxylin and eosin. The number of metastatic cancer nests was counted at 100× magnification using an inverted microscope (OLYMPUS, CKX53SF, Tokyo, Japan) for histological examination and metastasis evaluation. For all animal experiments, operators and researchers were blinded to the group assignments. All experimental procedures involving animals were performed in accordance with the guidelines for the care and use of laboratory animals and the institutional ethics guidelines.

### 2.9 Hematoxylin and eosin staining

Lungs were removed from mice and fixed with 4% paraformaldehyde for 12 h, embedded in paraffin, sectioned at a thickness of 4 μm with a microtome, and placed on slides. The paraffin sections were dewaxed at 65 °C for 1 h, after which the tissues were deparaffinized with turpentine, 90%, 75%, and 50% ethanol for further staining with hematoxylin and eosin. A neutral resin seal was then applied and photographed under a microscope.

### 2.10 Luciferase reporter assay

Luciferase reporter constructs were generated from the pMIR‐REPORT vector. The plasmids pMIR‐REPORT vector was purchased from Ambion (Austin, TX, USA) The wild‐type and mutant sequences of AATBC, containing miR‐1237‐3p binding sites, were synthesized and cloned into the pMIR‐REPORT vector. The sequences containing the putative miR‐1237‐3p and human PNN mRNA binding sites were amplified and cloned into the pMIR‐REPORT vector, and the sequences are shown in Table S2. Relative luciferase activity was measured by the Dual‐Luciferase Reporter Assay System (Promega, Madison, WI, USA) using SpectraMax^®^ iD3 microplate reader (Shanghai, China) (Xiao *et al*., 2019).

### 2.11 Western blotting

Total cell lysates were obtained using RIPA Lysis Buffer (Beyotime, Shanghai, China) supplemented with 1:25 Halt Phosphatase Inhibitor Cocktail (Roche, Shanghai, China), and protein concentration was determined using BCA Protein Assay Kit (Pierce, Grand Island, NY, USA). Protein samples were prepared to 20 μg per well, denatured in 100 °C for 10 min, separated by 10% SDS/PAGE, and then transferred to a PVDF membrane (Millipore, Shanghai, China). Membranes were immunoblotted with primary antibodies, anti‐PNN (Proteintech, Wuhan, China), anti‐E‐cadherin, anti‐N‐cadherin, anti‐ZEB1, anti‐ZEB2, anti‐SNAIL, or anti‐SLUG (CST, Danvers, MA, USA) antibodies. After washing, the blots were incubated with respective peroxidase‐conjugated secondary antibody (Proteintech, Wuhan, China). The blot was exposed to X‐ray film and developed using an enhanced chemiluminescence detection system (EMD Millipore, Burlington, MA, USA). GAPDH (CST, Danvers, MA, USA) served as the loading control.

### 2.12 Proteomics analysis

The UltiMate 3000 RSLCnano system coupled to the LTQ Orbitrap Velos Pro mass spectrometer (Thermo Scientific, Bremen, Germany) was used for proteomics analysis. Firstly, 5‐8F cells were transfected with siAATBC or the AATBC overexpression plasmid with their respective vector controls. At 48 h post‐transfection, the cells were lysed and peptides diluted with 0.1% trifluoroacetic acid, after which 5 μL sample was injected per assay. Next, the analytes were transferred to an analytical column and the proteins were identified using the proteome discoverer software (Thermo Scientific, Waltham, MA, USA) and matched to those in the Swiss‐Prot human database. The original files were used to search the UniProt KB/Swiss‐Prot database (release 2014_02). Peptide identification with false discovery rates < 1% (*q* < 0.01) was discarded. Four sets of the LC‐MS/MS data were normalized and filtered. Proteins ≥ 2 peptides and average area ratio‐fold changes ≥ 1.50 or ≤ 0.67 were considered as differentially expressed.

### 2.13 Immunoprecipitation assay

Nasopharyngeal carcinoma cells were transfected with the Flag‐PNN overexpression vector. The cells were harvested using GLB+lysis buffer (Beyotime) on ice. Protein A/G Magnetic Beads (Bimake, Houston, TX, USA) were incubated with primary antibody for 2 h at 25 °C on a rotator and then overnight at 4 °C. The magnetic bead–immune complex was washed 5–6 times with the lysis buffer, and the beads were resuspended in 6× protein loading buffer and boiled at 100 °C for 10 min to elute the bound protein from the beads. The eluted immune complexes were detected by western blotting.

### 2.14 Immunofluorescence

Nasopharyngeal carcinoma cell lines, 5‐8F, HNE2, or CNE2, were transfected with the PNN‐Flag overexpression vector on a six‐well plate. The cells were fixed with 4% paraformaldehyde for 40 min at 25 °C, treated with 0.3% Triton X‐100 at 37 °C for 30 min, and blocked with 5% BSA for 1 h. The cells were incubated with anti‐Flag and anti‐ZEB1 antibodies overnight at 4 °C and then with secondary antibody for 1 h at 37 °C (He *et al*., 2016). After counterstaining for 10 min with DAPI, the cells were imaged under a confocal microscope (Ultra‐View Vox; Perkin‐Elmer, Waltham, MA, USA).

### 2.15 Statistical analysis

All statistical analyses were performed using the spss 13.0 (IBM Corp, Armonk, NY, USA) and graphpad 5 (GraphPad Software, San Diego, CA, USA) software programs. Data were presented as mean ± SD. Student's *t*‐test was used when the differences between groups were similar, and the Wilcoxon signed‐rank test was used when the differences between groups were not similar. Overall survival and recurrence‐free survival were calculated using Kaplan–Meier log‐rank test analysis. Tumor marker prognosis analysis was performed according to the REMARK reporting guidelines. *P* values < 0.05 were considered to be significantly different.

## 3 Results

### 3.1 AATBC was highly expressed in NPC and associated with poor prognosis

To identify differentially expressed lncRNA in NPC, two NPC public microarray datasets (GSE64634 and GSE12452) were used to perform the significant analysis of microarray (SAM) (Wang *et al*., 2017, 2016). We observed 28 overlapping probe sets representing 24 differentially expressed lncRNA from two NPC datasets. Compared to the normal nasopharyngeal epithelia (NPE), 11 were highly expressed and 13 were downregulated in NPC. LOC284837, a lncRNA also designated AATBC, was noteworthy due to its role in regulating apoptosis in bladder cancer (Zhao *et al*., 2015). To confirm the expression of AATBC in NPC, two additional NPC gene expression datasets, GSE53819 and GSE68799, were analyzed. Results showed that AATBC was also highly expressed in both datasets (Fig. 1A). We then confirmed the overexpression of AATBC in 18 NPC biopsy samples by comparing with ten normal nasopharyngeal epithelial samples by quantitative real‐time PCR (qRT‐PCR) (Fig. 1B).

**Fig. 1:** AATBC was highly expressed in NPC tissues and associated with poor prognosis. (A) The expression of AATBC in NPC GEO datasets (GSE64634, GSE12452, GSE53819, and GSE68799). Error bars represent the standard deviation of the mean. *P < 0.05; ***P < 0.001. (B) The expression of AATBC was measured in NPC and NPE biopsies by qRT‐PCR, and β‐actin is used as endogenous control. Error bars represent the standard deviation of the mean. **P < 0.01. (NPE, nontumor nasopharyngeal epithelial tissue, *n* = 10; NPC, nasopharyngeal carcinoma tissue, *n* = 18). (C) Representative images of AATBC expression in NPC and NPE tissues by ISH. The pictures were captured at 200× (scale bars = 50 μm) and 400× (scale bars = 20 μm) magnifications. (D) Statistical analysis of ISH in 34 cases of NPE and 101 NPC biopsies. (E) Kaplan–Meier analysis of the correlation between AATBC expression and overall survival of NPC patients.

To further assess the AATBC expression in NPC tissues, *in situ* hybridization was performed in 101 NPC and 34 NPE paraffin sections using specific AATBC probes (Fig. 1C). The data indicated that the expression of AATBC was higher in NPC tissues compared to NPE tissues (Fig. 1D and Table S1). Survival analysis demonstrated that higher AATBC expression was correlated with poor overall survival in NPC patients (Fig. 1E). However, no correlation was observed between AATBC expression and clinical–pathological features of NPC patients, such as gender, age, smoking, histological type, pathological stage, tumor size (T stages), lymph‐vascular invasion (N stages), or relapse. These results suggest that high expression of AATBC was closely associated with NPC progression, and AATBC may serve as a powerful prognostic biomarker for NPC patients.

### 3.2 AATBC promoted NPC cell migration and invasion

To investigate the biological functions of AATBC in NPC, a siRNA targeting AATBC (siAATBC) was used to transiently knockdown its expression in NPC cell lines, 5‐8F, HNE2, and CNE2. The full‐length amplicon of AATBC was ligated to pcDNA3.1 expression plasmid to perform overexpression studies in NPC cells. The expression of AATBC was confirmed by qRT‐PCR analysis (Fig. S1A). Wound healing assay demonstrated that the migration ability of AATBC knock downed cells was significantly reduced. In addition, we observed that overexpression of AATBC enhanced the potential migration of NPC cells (Fig. 2A and Fig. S1B–D). In order to provide a better microenvironment for NPC cell growth to favor local adhesion, invasion, and distant metastasis of tumor cells, we established a 3D cell culture model to further explore the role of AATBC in cell invasion. The 3D invasion assay results showed that the NPC cell line, 5‐8F, formed invasive protrusion during the culture process; however, the invasive ability of spheroid cells was almost completely blocked when AATBC was knocked down. Compared to the control, AATBC re‐expressing cells had more invasive projections (Fig. 2B). Additionally, transwell Matrigel invasion assays showed that AATBC knockdown effectively inhibited tumor cell invasion, while overexpression of AATBC enhanced the invasion (Fig. 2C). These data indicate that AATBC promotes NPC cell migration and invasion *in vitro*.

**Fig. 2:** The biological functions of AATBC. (A) Would healing assays were monitored at 0, 12, and 24 h in AATBC knocked down or overexpressed NPC cells. The gap distance was showed as mean ± SEM of three independent experiments. Statistical significance is evaluated by *t*‐test. **P < 0.01; ***P < 0.001. (B) AATBC promoted invasiveness in 5‐8F spheroid clones and the formation of filopodia in 3D cell culture model. The black arrow indicates protrusions formed on the surface of the spheroid (top), scale bars = 50 μm. The graphs represent the quantification of invasive and noninvasive spheroid types in siAATBC and the AATBC‐overexpressing cells. (C) Transwell Matrigel assays were performed in NPC cells transfected with siAATBC and the AATBC overexpression vector with their respective empty vector controls. The relative proportion of invading cells in each field is shown as mean ± SEM of three independent tests. Statistical significance is evaluated by *t*‐test, **P < 0.05; **P < 0.01. (D) Bright‐field images of metastatic nodules in the lung tissues of mice, *n* = 6. (E) Significant metastases were visible in the lungs of all the three groups of mice, and arrows indicate colonies of lung tumor cells. (F) Graph representing the number of metastatic nodules observed in nude mice. Data presented as mean ± SEM (each data point represents a nude mouse, *n* = 6). **P < 0.01; ***P < 0.001. (G) The microscopic images of mouse lung biopsies stained by hematoxylin and eosin; the rectangular box represents the clusters of micrometastatic cells in the mouse lung. The pictures were captured at 100× (scale bars = 100 μm), 200× (scale bars = 50 μm), and 400× (scale bars = 20 μm) magnifications.

To confirm the functions of AATBC *in vivo*, 5‐8F cells transfected with the AATBC overexpression plasmid, siAATBC, or the empty vector were intravenously injected into the nude mice via the tail vein (6 mice per group). The mice were sacrificed, and the morphological changes in their lungs were observed after 8 weeks (Fig. 2D). Compared to the control group, the metastatic lesions at the lung surface were more abundant in the AATBC overexpression group than the NC group, while the metastatic nodules were less in AATBC knockdown group compared to the control (Fig. 2E,F). Hematoxylin–eosin (HE) staining of the lung tissue sections confirmed the observed morphological features (Fig. 2G). These observations hint the role of AATBC in promoting metastasis.

### 3.3 AATBC promoted NPC migration and invasion through PNN

To elucidate how AATBC promotes NPC migration and invasion, we constructed the proteomic profiles of 5‐8F cells transfected with the overexpression AATBC vector or siAATBC with their respective controls, using the liquid chromatography‐tandem mass spectrometry (LC‐MS/MS) strategy. A total of 205 differentially expressed proteins were detected after overexpression/knockdown of AATBC. Among them, 94 proteins were upregulated and 111 were downregulated. We also performed a correlation analysis to find the genes, which were highly correlated with AATBC in the NPC biopsy microarray data. There were 18 positively correlated genes and 25 negatively correlated genes with respect to the expression of AATBC in both the datasets, GSE64634 and GSE12452. LncRNA bind directly miRNA to act as sponges and neutralize the inhibitory effects of miRNA on their target mRNA. To elucidate whether AATBC serves as miRNA sponges, we focused on five proteins (genes), including PNN, ERP44, OLA1, SF3B3, and ITGB1, which were significantly upregulated by AATBC in 5‐8F cell line and the NPC microarray data (Fig. 3A). Among the five proteins, only PNN was confirmed to be positively regulated by AATBC in all the three NPC cell lines (5‐8F, HNE2, and CNE2) at both transcriptional and translational levels by qRT‐PCR (Fig. 3B,C) and western blotting analysis, respectively (Fig. 3D). Figure S2A indicated that PNN was upregulated in NPC and its expression was positively correlated with that of AATBC.

**Fig. 3:** Identification of proteins regulated by AATBC. (A) The differentially expressed proteins regulated by AATBC as determined by LC‐MS/MS, which mRNA were also positively correlated with AATBC in NPC biopsies. (B) qRT‐PCR analysis was used to validate the selected genes in 5‐8F, HNE2, and CNE2 cell lines. Data were presented as mean ± SEM of three independent tests. Student's *t*‐test was used in two groups. *P < 0.05; **P < 0.01; ***P < 0.001; and ****P < 0.0001. (C) qRT‐PCR analysis demonstrated PNN expression in NPC cells upon silencing or overexpressing AATBC. GAPDH was used as endogenous control. Data were presented as mean ± SEM of three independent tests. Statistical significance is evaluated by Student's *t*‐test. **P < 0.01; ***P < 0.001. (D) Western blotting analysis demonstrated PNN expression in NPC cells upon silencing or overexpressing AATBC. GAPDH was used as endogenous control.

PNN, a desmosome‐associated protein, plays a vital role in regulating epithelial cell–cell adhesion. Wound healing and transwell assays showed knockdown of PNN reduced migration and invasion potentials in NPC cells, while overexpression of PNN showed antagonistic effects (Fig. 4A,B and Fig. S2B,C). The migration and invasion abilities of NPC cells after AATBC knockdown were rescued when PNN was overexpressed. Also, the migration and invasion abilities of AATBC‐overexpressed NPC cells were reduced upon PNN knockdown (Fig. 4C,D and Fig. S3A,B). These results indicated that AATBC‐mediated NPC migration and invasion was modulated by PNN.

**Fig. 4:** AATBC promotes NPC cell migration and invasion through PNN. (A) The expression of PNN was detected by qRT‐PCR analysis in 5‐8F, HNE2, and CNE2 cells after transfection with siPNN or the PNN‐Flag vectors. β‐actin was used as endogenous control. Data were presented as mean ± SEM of three independent tests. Statistical significance is evaluated by Student's *t*‐test. *P < 0.05; **P < 0.01; ****P < 0.0001. (B) The expression of PNN was detected by western blotting analysis in 5‐8F, HNE2, and CNE2 cells after transfection with siPNN or the PNN‐Flag vectors. GAPDH was used as endogenous control. (C) The migration ability of 5‐8F cells was measured by scrape motility assays. Representative images showing the scratch widths at 0, 12, and 24 h, scale bars = 200 μm. The gap distance was showed as mean ± SEM of three independent experiments. Statistical significance is evaluated by *t*‐test. **P < 0.01; ***P < 0.001; and ****P < 0.0001. (D) Transwell assay was used to evaluate the invasive ability of NPC cells. Scale bars = 200 μm. The relative proportion of invading cells in each field were shown as mean ± SEM of three independent experiments. Statistical significance is evaluated two‐tailed Student's *t*‐test. **P < 0.01; ***P < 0.001.

### 3.4 AATBC acted as a ceRNA and interacted with miR‐1237‐3p

To identify the miRNA that might play a role in the AATBC‐PNN regulatory network in NPC, we predicted the miRNA binding sites in the AATBC full RNA sequence using different bioinformatics tools (RegRNA2.0, RNAhybrid, RNA22V2, and PITA). Three miRNA including miR‐1237‐3p, miR‐885‐3p, and miR‐638 were predicted to bind AATBC with low minimum free energy. The data of qRT‐PCR showed that AATBC downregulated the expression of miR‐1237‐3p but not miR‐885‐3p and miR‐638 consistently in all the three NPC cell lines, 5‐8F, HNE2, and CNE2 (Fig. 5A). Hence, we selected miR‐1237‐3p for further investigation. The data of qRT‐PCR indicated miR‐1237‐3p mimics reduced the expression of AATBC and PNN and miR‐1237‐3p inhibitors increased their expression in all three NPC cell lines (Fig. 5B,C). These results indicate that AATBC and PNN were negatively regulated by miR‐1237‐3p in NPC cells.

**Fig. 5:** AATBC functioned as a competing endogenous RNA to regulate PNN expression by sponging miR‐1237‐3p. (A) The expression of microRNA was detected by qRT‐PCR analysis upon transfection with siAATBC or the AATBC overexpression vector. Data were presented as mean ± SEM of three independent tests. Statistical significance is evaluated Student's *t*‐test. *P < 0.05; **P < 0.01; ***P < 0.001. (B) qRT‐PCR analysis of AATBC and PNN expression in NPC cells treated with miR‐1237‐3p inhibitor or mimics. Data were presented as mean ± SEM and three independent experiments. Statistical significance is evaluated by Student's *t*‐test. *P < 0.05; **P < 0.01; ***P < 0.001; and ****P < 0.0001. (C) PNN expression was detected in NPC cell lines (5‐8F, HNE2, and CNE2) transfected with the inhibitor or mimics of miR‐1237‐3p by western blotting using anti‐PNN antibody and normalized to GAPDH. (D) The sequences of the wild‐type (WT) and mutant (MT) AATBC were designed based on the predicted binding sites of miR‐1237‐3p. (E) Luciferase activities were measured in NPC cells co‐transfected with the AATBC‐WT or MT luciferase reporters and inhibitors or mimics of miR‐1237‐3p. Renilla luciferase activity was measured to normalize the transfection efficiency across the samples. Three independent experiments were performed to confirm the results. Data were presented as mean ± SEM. Statistical significance is evaluated by *t*‐test. *P < 0.05; **P < 0.01; ***P < 0.001. (F) Schematic diagram of the binding site of miR‐1237‐3p on the PNN 3′‐UTR. (G) Luciferase activities were detected in NPC cells after co‐transfection with the WT or MT reporters of PNN 3′‐UTR and miR‐1237‐3p inhibitor or mimics. Data were presented as mean ± SEM of three independent tests. Statistical significance is evaluated by *t*‐test. *P < 0.05; **P < 0.01; ***P < 0.001.

In order to confirm whether miR‐1237‐3p directly binds to the AATBC sequence and the PNN 3′‐UTR, we constructed luciferase reporter vectors, which possessed wild‐type (WT) or mutant (MT) sequences of the miR‐1237‐3p binding site on the AATBC sequence or the 3′‐UTR of PNN (Fig. 5D). The data showed that transfection of miR‐1237‐3p inhibitors induced the luciferase activity of the AATBC‐WT reporter, but not the mutant AATBC reporter. On the other hand, transfection of miR‐1237‐3p mimics reduced the luciferase activity of the AATBC‐WT reporter (Fig. 5E), suggesting that miR‐1237‐3p binds to AATBC through this site.

The WT and MT luciferase reporters of PNN were also constructed according to the binding site of miR‐1237‐3p to the 3′‐UTR of PNN (Fig. 5F). Luciferase assay showed that miR‐1237‐3p inhibitors increased the luciferase activity of the PNN 3′‐UTR WT sequence (pMIR‐WT), while the luciferase activity of the mutant PNN 3′‐UTR vector remained unchanged. Likewise, transfection with miR‐1237‐3p mimics had an opposite effect on the PNN 3′‐UTR luciferase activity (Fig. 5G). These results suggest that PNN was a target gene of miR‐1237‐3p and AATBC might act as a molecular sponge to facilitate the binding of miR‐1237‐3p with PNN.

### 3.5 miR‐1237‐3p was downregulated in NPC and inhibited cell migration and invasion

Next, we analyzed the microRNA expression profiling dataset GSE73460 and found that miR‐1237‐3p was downregulated in NPC clinical samples when compared with NPE (Fig. 6A). Wound healing and transwell invasion experiments demonstrated that transfection of miR‐1237‐3p inhibitors promoted NPC cell migration and invasion and miR‐1237‐3p mimics had an opposite effect in 5‐8F, HNE2, and CNE2 cell lines (Fig. 6B–D and Fig. S4A,B). Taken together, these results indicate that miR‐1237‐3p promoted NPC cell migration and invasion.

**Fig. 6:** miR‐1237‐3p was downregulated in NPC and inhibited cell migration and invasion. (A) miR‐1237‐3p was lowly expressed in 62 NPC tissues compared with 6 NPE tissues. Error bars represent the standard deviation of the mean. Statistical significance is evaluated by *t*‐test. ****P < 0.0001. (B) The expression of miR‐1237‐3p was detected by qRT‐PCR following transfection of NPC cells with miR‐1237‐3p inhibitors or mimics. Data were presented as mean ± SEM of three independent experiments. Statistical significance is evaluated by two‐tailed Student's *t*‐test. **P < 0.01; ***P < 0.001; ****P < 0.0001. (C) The migration ability was measured in 5‐8F cells after transfection with miR‐1237‐3p inhibitors or mimics using scrape motility assays. The gap distance was shown as mean ± SEM of three independent experiments. Statistical significance is evaluated by two‐tailed Student's *t*‐test. **P < 0.01; ***P < 0.001. (D) Cell invasion was analyzed in three NPC cells after transfection with miR‐1273‐3p mimics or inhibitors. The relative proportion of invading cells in each field is shown at the right as mean ± SEM of three independent experiments, scale bars = 200 μm; **P < 0.01; ***P < 0.001; ****P < 0.0001.

### 3.6 PNN regulated the activity of E‐cadherin through interacting with ZEB1

PNN regulates epithelial cell adhesion by binding to the E‐box 1 core sequence of the E‐cadherin gene promoter (Alpatov *et al*., 2004). A previous study also indicated that ZEB1 binds to the E‐box of the E‐cadherin promoter to modulate its gene expression (Singh *et al*., 2011). Hence, we hypothesized that PNN may form a complex with ZEB1 to regulate the promoter of E‐cadherin. Our immunoprecipitation studies showed an interaction between PNN and ZEB1 proteins in all three cell lines (Fig. 7A). Immunofluorescence staining also indicated colocalization of PNN and ZEB1 in three NPC cell lines (Fig. 7B). These results indicate that PNN might accelerate NPC migration and invasion by interacting with ZEB1.

**Fig. 7:** PNN regulated the activity of E‐cadherin through interacting with ZEB1. (A) Co‐IP experiment was detected the interaction between PNN and endogenous ZEB1 in NPC cells transfected with the PNN‐Flag vector. (B) Colocalization of PNN and ZEB1 proteins in 5‐8F, HNE2, and CNE2 cells. DAPI stained nuclei: blue; anti‐Flag‐PNN: red; anti‐ZEB1: green; merged images represent the stack of DAPI, Flag, and ZEB1 signals; scale bars = 29 μm.

### 3.7 AATBC promoted the EMT progress through PNN

To probe whether AATBC regulates the EMT progress through PNN, we knocked down AATBC or PNN to observe the changes in the expression of epithelial and mesenchymal markers. The expression of E‐cadherin was reduced, and the expression of N‐cadherin, SNAIL, SLUG, ZEB1, and ZEB2 proteins was induced in NPC cells after siAATBC or siPNN transfection (Fig. 8A,B). Additionally, overexpression of AATBC and PNN reduced E‐cadherin expression and enhanced N‐cadherin, SNAIL, SLUG, ZEB1, and ZEB2 expression (Fig. 8B). These results indicated that AATBC might regulate the EMT progress in NPC through PNN.

**Fig. 8:** AATBC promoted the EMT progress through PNN protein. (A) The transcriptional levels of E‐cadherin were detected by qRT‐PCR in NPC cell lines after knockdown or overexpression of AATBC and PNN. Data were presented as mean ± SEM of three independent experiments. Statistical significance is evaluated by two‐tailed Student's *t*‐test. *P < 0.05; **P < 0.01; ***P < 0.001. (B) Expression analysis of the EMT pathway‐associated proteins (E‐cadherin, N‐cadherin, ZEB1, ZEB2, SNAIL, and SLUG) by western blot in NPC cell lines after knockdown or overexpression of AATBC and PNN. GAPDH was used as an endogenous control.

## 4 Discussion

Nasopharyngeal carcinoma is one of the most aggressive cancer in which metastasis is reported to be the cause of mortality (Fan *et al*., 2019a; Wu *et al*., 2019b; Wu *et al*., 2020 ). The molecular mechanism governing NPC metastasis is little known (Tang *et al*., 2018b). Using the human transcriptome microarray analysis, we identified a lncRNA, AATBC, which was highly expressed in NPC samples and its expression positively correlated with NPC patients' prognosis.

Until now, only one paper had reported that AATBC can promote proliferation and inhibit apoptosis in bladder cancer. It has been found that inhibition of AATBC induced p‐JNK and reduced NPF2 (NF‐E2‐related factor 2) while activating the expression of caspase‐9 and caspase‐3 to promote apoptosis in bladder cancer cells (Zhao *et al*., 2015). Next, we examined whether AATBC regulated apoptosis in NPC cells. Unlike in bladder cancer cells, AATBC did not inhibit apoptosis but rather promoted migration and invasion potential of NPC cells. Therefore, we deduced that AATBC may exert different functions on bladder cancer compared to NPC.

LncRNA act as a molecular ‘sponge’ to adsorb miRNA to form a lncRNA–miRNA axis. It possesses ceRNA characteristics and participates in the regulation of various cellular signaling pathways (Bo *et al*., 2018; He *et al*., 2017; Zhong *et al*., 2018). LncRNA, AFAP1‐AS1, acts as a ceRNA of miR‐423‐5p and regulates Rho/Rac pathway to promote NPC (Lian *et al*., 2018). LncRNA KRTAP5‐AS1 and TUBB2A regulate CLDN4 expression by acting as a sponge to adsorb miR‐596 or miR‐3620‐3p in gastric cancer (Song *et al*., 2017). LncRNA MIR100HG acts as ceRNA for miR‐100 and miR‐125b to regulate Wnt/β‐catenin signaling, thus contributing to cetuximab resistance in colorectal cancer (Lu *et al*., 2017; Mo *et al*., 2019b). In this study, we found that AATBC acts as a ceRNA to regulate the expression of PNN and aided the EMT progress and the metastasis of NPC by binding to miR‐1237‐3p.

Mass spectrometry results revealed that PNN, a desmosome‐associated protein, was upregulated by AATBC and highly expressed in NPC tissues. Further, our data showed that PNN interacted with the transcription factor ZEB1 to promote the ZEB1‐mediated EMT process of NPC cells, leading to PNN‐dependent repression of E‐cadherin to regulate epithelial cell–cell adhesion (Alpatov *et al*., 2004). Due to the specificity of tumors, we speculated that PNN and ZEB1 combined to form a more stable complex and promoted the expression of ZEB1. However, the specific mechanism associated with this action is yet to be determined and further studies are needed to more completely investigate these regulatory networks (Zhang *et al*., 2018).

In this study, we employed mass spectrometry to screen differentially expressed proteins by AATBC. There were 205 proteins that were found to be significantly regulated by AATBC. It is worthy to elucidate how these proteins were regulated by AATBC as well as the mechanism to promote NPC metastasis. LncRNA can regulate the transcription and post‐transcriptional activity of target genes to exert distinctive biological functions in the pathogenesis of cancer. In fact, certain lncRNA can directly bind to target proteins and regulate their localization (Duan *et al*., 2019; Xia *et al*., 2019), stabilization, and post‐translational modifications (Fan *et al*., 2017). Hence, lncRNA employ various molecular interaction models to influence the initiation, progression, and metastasis of cancer (Deng *et al*., 2018; Fan *et al*., 2019c).

## 5 Conclusions

This study deciphers the key molecular functions of AATBC, an upregulated lncRNA in NPC. Future studies may serve to elucidate potential avenues for utilizing AATBC as a prognostic biomarker for early detection of NPC. Moreover, the AATBC/miR‐1237‐3p/PNN axis may function as a significant pathway that promotes NPC metastasis and, therefore, may be a novel diagnostic and therapeutic target in NPC patients.

## Conflict of interest

The authors declare no conflict of interest.

## Author contributions

ZZ conceived and designed the project. TT, LY, YC, MW, SZ, ZG, FX, YH, and YZ conducted the experiments and acquired the data. QL, BX, MZ, CG, XL, YL, WX, and GL analyzed the data. ZZ, WX, and TT wrote the paper. All authors approved the final manuscript.

## Supporting information


**Fig. S1.** AATBC reinforced the migration and invasion capacities of NPC cells *in vitro*. (A) qRT‐PCR was used to detect the silencing and overexpression efficiencies of AATBC in NPC cell lines. Data were presented as mean ± SEM of three independent experiments. Statistical significance is evaluated by t‐test. **, *p* < 0.01; ***, *p* < 0.001; ****, *p* < 0.0001. (B–D) The migration ability of NPC cells (5‐8F, HNE2, and CNE2) after knockdown or re‐expression of AATBC was measured by wound healing assays.

**Fig. S2.** PNN promoted NPC cells migration and invasion. (A) PNN was highly expressed in 31 NPC tissues compared with 10 NPE tissues (left panel); Error Bars represent the standard deviation of the mean, ***, *p* < 0.001. The expression of AATBC was positively correlated with PNN in the NPC dataset GSE12452 (right panel). (B) The migration ability of NPC cells was investigated after treatment with siPNN or the PNN‐Flag vector using scrape motility assays. Images were acquired at 0, 12, and 24 h. The gap distance was showed as mean ± SEM of three independent experiments, two‐tailed Student's t‐test, *, *p* < 0.05; **, *p* < 0.01; ***, *p* < 0.001; ****, *p* < 0.0001. (C) Transwell invasion assays were performed in NPC cells (5‐8F, HNE2, and CNE2) after knockdown or overexpression of PNN. The relative proportion of invading cells were showed as mean ± SEM (n = 3 independent tests), two‐tailed Student's t‐test. **, *p* < 0.01; ***, *p* < 0.001.

**Fig. S3.** PNN promoted NPC cells migration and invasion. (A) PNN was highly expressed in 31 NPC tissues compared with 10 NPE tissues (left panel); Error Bars represent the standard deviation of the mean, ***, *p* < 0.001. The expression of AATBC was positively correlated with PNN in the NPC dataset GSE12452 (right panel). (B) The migration ability of NPC cells was investigated after treatment with siPNN or the PNN‐Flag vector using scrape motility assays. Images were acquired at 0, 12, and 24 h. The gap distance was showed as mean ± SEM of three independent experiments, two‐tailed Student's t‐test, *, *p* < 0.05; **, *p* < 0.01; ***, *p* < 0.001; ****, *p* < 0.0001. (C) Transwell invasion assays were performed in NPC cells (5‐8F, HNE2, and CNE2) after knockdown or overexpression of PNN. The relative proportion of invading cells were showed as mean ± SEM (n = 3 independent tests), two‐tailed Student's t‐test. **, *p* < 0.01; ***, *p* < 0.001.

**Fig. S4.** miR‐1237‐3p inhibited the migration of NPC. Scrape motility assays were used to explore the migration ability of NPC cells (HNE2 (A) and CNE2 (B)) transfected with miR‐1237‐3p inhibitors or mimics. The data are shown as mean ± SEM, n = 6. Statistical significance is evaluated by t‐test. *, *p* < 0.05; **, *p* < 0.01; ***, *p* < 0.001.

**Table S1.** The clinical information and the expression of AATBC in 101 paraffin‐embedded NPC biopsies measured by *in situ* hybridization.

**Table S2.** Primers used for qRT‐PCR and constructions or siRNA.
